# Ultrasound-Facilitated Catheter-Directed Thrombolysis via Dual Right Upper Extremity Venous Access Into the Basilic Vein in a Case of Submassive Pulmonary Embolism

This article has been retracted.

**DOI:** 10.7759/cureus.12545

**Published:** 2021-01-07

**Authors:** Ahmed Elkhouly, Derek Enos, Justin Fox

**Affiliations:** 1 Internal Medicine, St. Francis Medical Center, Trenton, USA; 2 Cardiology, St. Francis Medical Center, Trenton, USA

**Keywords:** submassive pulmonary embolism, catheter-directed thrombolysis, ultrasound guided catheter directed thrombolysis, ekos

## Abstract

Traditionally, massive, life-threatening pulmonary embolism (PE) has been treated with systemic thrombolytic therapy while submassive and smaller acute PEs have been treated with systemic anticoagulation therapy. Given that thrombolytic therapy is associated with the risk of life-threatening complications including intracranial hemorrhage, it has not been routinely used or recommended for submassive PEs. In 2017, the Food and Drug administration (FDA) approved ultrasound-facilitated catheter-directed thrombolysis (USCDT) for acute massive and sub-massive pulmonary embolism. USCDT has primarily been performed using jugular or femoral venous access. There have been isolated reports of USCDT performed through upper extremity venous access. We present a case of USCDT in a submassive PE patient with dual right upper extremity venous access where both sheaths were advanced into the basilic vein (due to anatomic variation). Based on recent clinical trial data suggesting that shorted duration USCDT is as effective as longer duration, tissue plasminogen activator (tPA) was infused in this case for 6 hours. This strategy for intervention can enhance patient comfort with USCDT therapy and can be particularly helpful in patients at high risk for access site complications and those unable to lie supine for the long duration of infusion therapy.

## Introduction

Pulmonary embolism (PE) was mentioned in the literature as early as the 1800s and was often associated with fatal outcomes. In 1960, a trial on the efficacy of systemic anticoagulation using intravenous heparin in pulmonary embolism showed a reduced mortality rate of 17% [1]. While the Centers for Disease Control and Prevention (CDC) estimates the yearly PE-related deaths in the United States at 60,000-100,000 [2], advanced imaging modalities, including computed tomography pulmonary angiography (CTPA) have drastically re-shaped PE diagnosis and prognosis. From 1998 to 2006, cases of pulmonary embolism detected in the US have nearly doubled without any change in mortality [3]. Massive (or high-risk) PE is a term used to describe patients with sustained hypotension (systolic blood pressure <90 mmHg for at least 15 minutes or those requiring inotropic support due to non-PE cause), pulselessness, or persistent profound bradycardia. Sub-massive (or intermediate risk) PE refers to those patients with acute PE without systemic hypotension but with evidence of either right ventricle (RV) dysfunction or myocardial necrosis. RV dysfunction is characterized by RV dilation, hypokinesis, or elevation of brain natriuretic peptide (BNP); myocardial necrosis is suggested by elevated troponin [4].

Patients presenting with sub-massive acute PE and impending right-sided heart failure usually benefit from systemic fibrinolytic therapy. Unfortunately, systemic fibrinolytic therapy has been associated with increased risk for major bleeding including intracranial hemorrhage and hemorrhagic stroke [5]. The advantage of percutaneous intervention using ultrasound-facilitated catheter-directed thrombolysis (USCDT) with low-dose thrombolytic infusion for a shorter period of time is successful local treatment delivery with noted reduction in the clot burden and minimal systemic side effects [6-8]. There has been a report of using the superficial veins of the upper extremity to place the two infusion catheters into cephalic and basilic vein separately to treat a patient with acute saddle PE. In our case, due to anatomical variation in the patient’s upper extremity venous system, both catheters ended up inside the basilic vein without any hematoma at the site of insertion. The OPTALYSE PE trial demonstrated that shorter durations (2-8 hours) of USCDT demonstrate similar benefits in terms of reducing right heart strain as longer durations (12-24 hours) [9]. In this case, we successfully utilized a lower dose of tissue plasminogen activator (tPA) for 6 hours, which enhanced patient comfort.

## Case presentation

We present a 33-year-old male patient with past medical history significant for morbid obesity, hypertriglyceridemia, protein S deficiency and lower extremity deep venous thrombosis (DVT) six years prior who presented with the acute onset of severe dyspnea and substernal pressure like exertional chest pain. The pain was non-radiating, not associated with nausea, vomiting or diaphoresis and alleviated partially with rest. On physical examination, he had a blood pressure of 124/60 mmHg, pulse of 118 beats/min, respiratory rate of 12 breaths/min and oxygen saturation of 97% on 2-liter nasal cannula. He was obese and demonstrated vesicular breathing on chest auscultation, normal heart sounds without any significant murmurs on cardiac examination and chronic left lower extremity edema secondary to his old DVT. The remainder of his physical examination was unremarkable. Patient’s surgical, social, and family histories were unremarkable.

Laboratory findings were significant for elevated D-dimer of 4908 ng/dL (<250 ng/dL), Troponin T less than 0.02 ng/mL (<0.04 ng/mL), partial thromboplastin time (PTT) 27.9 seconds, white blood count of 11.4 (4.5-11), hemoglobin of 13.6 g/dL (13.5-17.5 g/dL) and platelets of 237 (150-450). Blood urea nitrogen of 12 mg/dL (7-20 mg/dL) and creatinine of 0.8 mg/dL (0.8-1.2 mg/dL). The remainder of his blood work was unremarkable. An initial electrocardiogram (EKG) demonstrated normal sinus rhythm at 87 beats/min without any significant ST-T wave changes. There were no electrocardiographic signs for possible right ventricular (RV) strain. Due to a high suspicion of pulmonary embolism, the patient underwent CT pulmonary arteriography that showed large bilateral central pulmonary embolism that extended distally, principally into both the left and right lower lobe branches (Figure 1). Bedside echocardiography showed normal left ventricular size and systolic function with ejection fraction of 60-65%. There was mild to moderate RV dilatation with mildly reduced RV systolic function associated with systolic and diastolic septal flattening consistent with RV pressure and volume overload. In the emergency department, the patient demonstrated worsening tachycardia and hypoxia with worsening of his symptoms.

**Figure 1:** CT pulmonary arteriography showing large bilateral pulmonary embolism (white arrows).

In the setting of this patient’s submassive pulmonary embolism, the decision was made to treat with USCDT, utilizing bilateral pulmonary artery infusion catheters. Due to his body habitus and large cubital veins, upper extremity venous access was chosen. Before prepping the right arm in the cardiac catheterization laboratory, two 20G Angiocath peripheral intravenous (PIV) catheters were placed in the right antecubital fossa, one medial and one lateral. The intention was to advance one infusion catheter via the cephalic vein and the other via the basilic vein. Limited contrast venography performed via each of the PIVs demonstrated that the medial PIV was placed in the basilic vein and the lateral PIV was in a small antecubital vein that appeared to drain more directly to the larger basilica vein. The vein connection to the relatively diminutive cephalic vein involved sharp angulation (Figure 2). We decided to proceed with the procedure through these two access sites with the plan to direct both sheaths into the basilic vein.

**Figure 2:** Panel A demonstrates contrast venography through the medial PIV and Panel B demonstrates contrast venography through the more lateral PIV. The images reveal the medial PIV to be placed in the basilic vein (black arrow) in panel A. The lateral IV is revealed to be placed in a small antecubital branch (orange arrow) that drains bidirectionally into a diminutive cephalic vein (red arrow) and larger basilic vein (black arrow) in panel B. PIV: Peripheral intravenous

The right arm was prepped and draped sterilely. The medial PIV was exchanged over a guidewire for a 6F slender glide sheath (Terumo Medical, Tokyo, Japan). The lateral PIV was exchanged in the same technique. There was no difficulty or resistance noted in advancing the two introducer sheaths into the right basilic vein. Through the more medial sheath we performed a right heart catheterization with a 5F Swan Ganz catheter, demonstrating right atrial pressure of 14 mmHg, pulmonary artery pressure of 55/26 mmHg and pulmonary capillary wedge pressure of 21 mmHg. The Swan Ganz catheter was exchanged over a V18 wire for a 12cm USCDT infusion catheter (Ekosonic Endovascular System, Boston Scientific, Marlborough, MA), placed in the left lower lobe pulmonary artery branch. This sequence of steps was repeated through the more lateral sheath with an infusion catheter placed in the right lower lobe pulmonary artery branch (Figure 3). tPA was delivered at the rate of 1 mg/hr for each lung with total of 12 mg of tPA over 6 hours. After 6 hours, catheters and sheaths were removed and the patient’s symptom of dyspnea at rest was resolved.

**Figure 3:** Fluoroscopic image of the two 6F infusion catheters (Ekosonic Endovascular System, Boston Scientific), in both pulmonary arteries.

## Discussion

Ultrasound-facilitated catheter-directed thrombolysis (USCDT) is a minimally invasive technique for intravascular thrombolysis, in this case for use in the pulmonary arteries for sub-massive bilateral pulmonary emboli. The mechanism of action is based on an acoustic field created by the ultrasonic core of the catheter, leading to thrombolysis through driving the anticoagulant drug deeper into the clot and unwinding the fibrin to expose plasminogen receptor sites. USCDT treatment utilizing the Ekosonic Endovascular System has been shown to be clinically superior to anticoagulation with heparin alone in patients suffering from intermediate risk and massive PE. In both ULTIMA [7] and SEATTLE II trials [8], the Ekosonic Endovascular System was superior in reversing right ventricular enlargement with improvement of RV/LV ratio, pulmonary artery pressure, cardiac index, and patient symptoms. Both trials used tPA over 12 to 24 h at total doses of 20 to 24 mg for acute pulmonary embolism. More recently, the OPTALYSE PE [10] trial showed that tPA at a lower total doses (4 to 12 mg per lung) and with shorter period infusion duration from 2 to 6 hours had similar results as the previous trials with reduction in right ventricular-to-left ventricular diameter ratio and improvement in the patient’s symptoms.

Common femoral vein or internal jugular vein access has been used for catheter-directed thrombolysis most frequently [6-8]. In SEATTLE II, the right femoral, left femoral, and right internal jugular veins were chosen as access sites for 63.7%, 21.9%, and 11.2% of cases, respectively [8]. In the PERFECT registry, approximately 6% of patients experienced minor or moderate bleeding including access site hematoma [6]. Access-related major bleeding defined as moderate or severe/life threatening bleeding was reported in approximately 5% of cases. There was a link between bleeding complications and access site attempts. The incidence of access site bleeding was 25.9% when multiple access attempts were made compared to only 4.0% when access was obtained on a single attempt [8]. A patient’s body habitus, specifically if obese, can impact the accessibility of the femoral or jugular veins, increasing the likelihood of multiple access attempts which in turn will increase the risk for hematoma. By utilizing superficial upper extremity venous access, complications such as hematoma, pseudoaneurysm, AV fistula, and pneumothorax are significantly reduced [10]. In addition, superficial upper extremity venous access for PE thrombolysis is more convenient for the patient with the ability to sit upright, change position, and even stand, making it yet another added benefit compared to the femoral access.

There was one case reported where USCDT catheters were introduced into the superficial veins of the right upper extremity with bilateral pulmonary artery catheters advanced through the cephalic and basilic veins separately to deliver tPA for 12 hours [11]. In our case report due to anatomical variation in the patient upper extremity venous anatomy both catheters ended in the basilic vein.

In our case due to the patient’s body habitus and obesity, we decided to proceed with upper extremity access to avoid multiple attempts in the femoral region. Due to anatomical variation of the patient right upper extremity venous system, both access sheaths were advanced into the basilic vein, without difficulty or complication. The arm was immobilized to avoid any catheter dislodgement and tPA was delivered for 6 hours with successful improvement in the patient’s symptoms.

## Conclusions

To enhance patient comfort and to limit the risk of access site complications, superficial venous access of the upper extremity through basilic and cephalic veins can be utilized for treating pulmonary embolism using thrombolytic infusion catheters. Performing venography through the peripheral intravenous catheters prior to placing the introducer sheath allows us to visualize the venous anatomy of the upper extremity prior to sheath insertion thus limiting the risk of local complications including hematoma. In addition, coupling upper extremity venous access with the strategy of using a lower dose and shorter duration of catheter directed thrombolytic therapy will enhance patient comfort and may reduce the risk of bleeding complications.
